The article "Electronic Sports Sustainable Development of Probing into Digital Games, Teenage Domestication, and Mutual Construction" was published in 2022. Journal: J Environ Public Health.

# Electronic Sports Sustainable Development of Probing into Digital Games, Teenage Domestication, and Mutual Construction

**DOI:** 10.1155/2022/6375787

**Published:** 2022-07-14

**Authors:** Peng Shao, Han Yu, Yujia Zhu, Junwei Wang

**Affiliations:** ^1^School of Humanities, Zhejiang University of Technology, Hangzhou 310051, China; ^2^School of Humanities, Tsinghua University, Beijing 100084, China; ^3^Zhejiang League College, Hangzhou 310051, China; ^4^School of Media and Law, NingboTech University, Ningbo 315000, China

## Abstract

The purposes is to investigate how digital games affect teenagers' physical and mental sustainable development and analyze the interactions and communications between teenagers and digital games using the domestication theory. *(1) Background*. A healthy mutual-domestication relationship is needed between teenagers and digital games. Digital games are expected to play a positive and decisive role, while parents and teachers should master the correct game literacy. *(2) Methods*. This study described the mutual domestication between them using interviews and questionnaires. *(3) Results*. Results demonstrate that digital games entering teenagers' lives are domesticated and marked with unique attributes caused by teenagers' different habits, during which parents and teachers are critical. In turn, digital games tame teenagers lifestyles and habits, becoming a popular social media among them. Spending excessive time and energy, teenagers will be addicted to digital games. *(4) Conclusions*. It can provide a reference for investigating the connection between teenagers and digital games.

## 1. Introduction

Digital games are implemented on digital devices and platforms. They are malleable and essential. Digital games have developed rapidly in the past few years. However, some groups, especially teenagers, can get addicted to games. Game addiction refers to the behavioral and mental status of individuals strongly obsessed with digital games due to the excessive time and energy spent on games. Digital games can shift the social ecology rather than simply providing entertainment [1].

Wong and Lam explored the relationship between teenagers' game behaviors and game addiction. They found that games could fulfill people's interest and help develop team cooperation. However, game addiction would result in emotional distress and even physical injury. Their work provided a basis for preventing game addiction [2]. Sadat-Shirazi et al. discovered that game addiction could lead to metabolic dysfunctions, and eventually physical damage [3]. Lin et al. investigated the connection between game quality and user perception as per game reviews on STEAM, a gaming platform [4]. Rachel believed that the gamer culture had grown into a “toxic culture” [5]. Federica et al. provided a systematic review on applying digital games to cognitive and emotional training in the adult population [6].

The article "Electronic Sports Sustainable Development of Probing into Digital Games, Teenage Domestication, and Mutual Construction" was published in 2022. Journal: J Environ Public Health.

Roger Silverstone put forward the domestication theory; afterward, Leslie Haddon and Maren Hartmann expanded its paradigm. Domestication is a concept that originated from biology; it originally reveals how human beings tame animals and plants [7]. Siles defined the association between users and recommendation algorithms using mutual domestication [8]. Bonchev et al. assessed the patterns of evolutionary trajectories and domestication history within the genus horde by REMAP markers [9].

Domestication in disciplines other than biology is defined as a cycle, namely, mutual domestication, during which each element is interdependent and complementary. Media testing is also a domestication process, interactive and synchronous rather than continuous. Mutual domestication occurs naturally through interaction [10, 11]. Domestication describes the acceptance, rejection, and use of media technologies as social behaviours based on social structures. Domestication of state-of-art technologies should include particular structures, users' values, and actual environments, pretty common in familial environments. Successfully domesticated technologies are practical tools accepted and trusted. Domestication emphasizes not only the use of technology but also the creation of an intermediary environment. Domestication believes that subjects like families and individuals have sociality; that is, they can exchange and interact with society.

Digital games have developed rapidly in recent years, penetrating a variety of social areas. Similarly, domestication can describe interactions and communications between teenagers and digital games. Hence, it applies to the research on digital games and mutual construction. Some researchers have proposed reverse domestication to explore media technology regulation. Li and Du pointed out that social media enriched the leisure time of college students and explored their impacts on procrastination. However, excessive time spent on social media could lead to Internet addiction [12]. Liu believed that reverse domestication was one of the most differentiated social media affecting the education of teenagers living in rural settings [13].

Meanwhile, some researchers have explored the dialectical relationship between technology and human beings using mutual domestication. Goulden took “smart home” as the example of platform capitalism. Results revealed family members' resistance due to the “interpersonal relationship data” generated by the Internet of Things interferes [14]. Therefore, mutual domestication does not define the motivation of information technology [15]. Regarding digital games, the domestication framework can investigate players' characteristics such as gender and age. Research on the collective domestication of digital games has broken the limitations of analyzing a single player's acting strategies. Studying team players and guilds reveals how the domestication of individual's acts in concert to produce compatible results [16]. To own a digital game, teenagers must possess electronic devices. However, devices that teenagers use to play digital games often belong to their parents [17].

The article "Electronic Sports Sustainable Development of Probing into Digital Games, Teenage Domestication, and Mutual Construction" was published in 2022. Journal: J Environ Public Health.

Game live-streaming has developed quickly in China. Professional players display how they play digital games via live broadcasts, while audiences can feel like playing the games together with the players they adore; moreover, the gratuity feature provided by live-streaming platforms can offer an extra income for professional players. Online interaction can promote offline cooperation; for example, Wang discovered that World of Warcraft players often enjoyed the game with their friends, roommates, and classmates together, forming online-offline communities [18]. However, the above works cannot reveal how games affect players. Digital games are unique intangible media that can switch between the public and private (offline and online). In the present study, the research objects possess diverse characteristics. On the one hand, digital games are intangible media attached to tangible media such as desktops, tablets, and smartphones. On the other hand, parents and teachers participate and affect the mutual domestication between digital games and teenagers. Hence, parents and teachers are included in the present study as well. The included research objects are surveyed with questionnaires and interviewed to investigate the mutual relationship between digital games and teenagers.

A review of recent works reveals a correlation between digital games and teenagers; nevertheless, how to quantitatively analyze such a correlation needs to be solved urgently [19]. In the present study, how digital games and teenagers affect each other is investigated, drawing on the domestication theory. Specifically, how such mutual influences affect society, the roles of parents, and teenagers in-between digital games and teenagers, and how can teachers and teenagers affect the domestication of digital games and teenagers are discussed and explained in detail. Therefore, the interactions and communications between digital games and teenagers are analyzed, and the roles of teachers and parents in the domestication process are investigated, to help teenagers master correct game literacy and promote a healthy relationship between teenagers and digital games.

The article "Electronic Sports Sustainable Development of Probing into Digital Games, Teenage Domestication, and Mutual Construction" was published in 2022. Journal: J Environ Public Health.

## 2. Theories and Methods

### 2.1. Game Literacy Education

In this study, we deem that game addiction of teenagers originates from the sense of belonging among peer groups. Children depend on their parents, while teenagers seek more socialization. In some cases, teenagers will feel isolated if they do not play any games because they have nothing in common with their peers. Digital games are regarded as a kind of bridge, which could connect different classes. As information technology develops at an unprecedented speed, growing in an era full of digital media, teenagers become aboriginals of digital culture. Computers, digital games, and the Internet have become teenagers' “living necessities.”

Digital literacy is the criterion for dividing the digital classes. On the one hand, game literacy is defined as the player's ability to actively participate in digital games and “control” the symbol systems of digital games. It represents a player's ability to combine gaming elements with social practices and output the combination results to the external environment. On the other hand, game literacy also refers to the ability to recognize, understand, experience, appreciate, determine, evaluate, design, and make games, that is, technical ability and literary accomplishment. Specifically, technical ability indicates a player's knowledge about games, gaming skills, and the ability to process, collect, and utilize the information for innovation. Literary accomplishment describes the player's mentality, moral cultivation, and critical ability.

Building social bonds is a “secret weapon” for capitals to keep the stickiness of players to the games they launched [20]. However, excessive attention to “team obligation” is unfavorable. If players cannot reflect on the online rules bound by interpersonal relationships and capital tendency, they will be “forced” to long-term games by technical intention, leading to another form of “game addiction.” In this regard, teenagers must receive game literacy education instead of banning them from games.

This study first proposes the game literacy theory; moreover, questionnaires are designed according to the recent works on digital games. Since parents and teachers face practical challenges in teenagers' game literacy education [21], home-school cooperated education is adopted.

### 2.2. Interview Plans

#### 2.2.1. Interview Content and Form

Interview refers to the direct contact and communication between the researchers and the interviewees, helping researchers understand interviewees' feelings and views, thereby acquiring the potential information needed [22]. Hence, we select interviews as the qualitative analysis approach. Because parents and teachers are vital in teenagers' growth, the interview focuses on teachers and parents, as well as game education professionals. The interview for parents plans to investigate is as follows: (1) games' influences on teenagers' daily situations, (2) whether they play digital games themselves, (3) the gaming atmosphere inside the family, and (4) their views on their children playing digital games.

The article "Electronic Sports Sustainable Development of Probing into Digital Games, Teenage Domestication, and Mutual Construction" was published in 2022. Journal: J Environ Public Health.

The interview for teachers plans to survey is as follows: (1) the academic performances of students from different grades who enjoy playing digital games, (2) the academic results of students in urban and rural areas who enjoy playing digital games, and (3) teachers' views and treatments for students who enjoy playing digital games on campus. The interview for game education professionals plans to explore the correlation between education and games. The interviews are finished via telephone or face-to-face conversations. During interviews, interviewers asked questions and adjusted the interview plans in real-time as per the answers of the interviewees. Each interview lasts for one hour. While all interviews are finished, the records are sorted, summarized and, and analyzed by content analysis. Finally, the interactive correlation between teenagers and digital games is discussed and analyzed based on the interview and questionnaire results.

### 2.3. Interview Sampling

We adopt two approaches to achieve the interview sampling. Firstly, snowball sampling is implemented in synchronization with the questionnaire. Six out of twenty teachers recommended by five schools are interviewed; background information considered includes gender, working years, course(s) responsible, and whether they are regular teachers or grade leaders who are aware of students and courses. Subsequently, considering gender, age, occupation, children's age, and whether working in other cities, six parents concerning about their children playing digital games are interviewed among 12 parents recommended by the six teachers. We got similar responses by the time we interviewed these 12 participants; hence, saturation was determined.

Second, purposive sampling is adopted, focusing on that the samples can accurately answer the questions rather than the sample size. Considering the recommendations of the interviewed teachers and the online and offline information, four professionals engaging in teenage game education are interviewed. Before the interview, they are informed of the research purposes and agree to accept the interview. Thy are as follows: (1) one teacher of an extracurricular activity center for teenagers, (2) one teenager programming teacher [13], (3) one game planner, and (4) one game self-media practitioner (with a Master's degree) to ensure the comprehensiveness of information.

The article "Electronic Sports Sustainable Development of Probing into Digital Games, Teenage Domestication, and Mutual Construction" was published in 2022. Journal: J Environ Public Health.

### 2.4. Research Samples

According to statistics, the Chinese game market is gradually saturated [19], exerting a negative impact on left-behind children. Jiangxi Province, located in midsouthern China, ranks 16th, 14th, and 21st in economic, education, and Internet development among 31 provinces and cities across China, respectively. Moreover, the number of migrant workers from Jiangxi rates top three in China, with an annual migrant population of 3.4 million, accounting for 7.25% of the total population [20, 21, 23]. We choose to perform the interview with teachers and parents from Huaqiao town (in Shangrao City) and Nanchang City, Jiangxi Province. Nanchang is the capital and the only second-line city in Jiangxi. The reform of state-owned enterprises in Huaqiao makes the problem of left-behind children prominent. Hence, selecting these two areas can maximize the effectiveness of the samples and take into account the urban-rural comparison.

### 2.5. Questionnaire Surveys

#### 2.5.1. Questionnaire Content and Form

Questionnaires investigate representative samples quantitatively [24]. In contrast, an interview is a qualitative approach, providing guiding opinions or suggestions on the questionnaire survey based on quantitative analysis. Since its results can be presented quantitatively, the questionnaire survey is objective and accurate. In this study, the criteria for assessing game addiction are the Clinical Diagnostic Criteria of Internet Addiction proposed by Tao Ran, Department of Medical Addiction, General Hospital of Beijing Military Region. These criteria are included in the game addiction section of the Diagnostic and Statistical Manual of Mental Disorders (DSM-5) by the American Psychiatric Association, marking that criteria formulated by Chinese scholars are recognized internationally in mental illness diagnosis for the first time, filling the gap in nonmaterial addictions and confirming that game addiction is a new disease that belongs to the category of mental illness diagnosis. This questionnaire aims to investigate the proportion of gamers among teenagers of different genders, places of growth, grades and academic results, and the characteristics of teenagers addicted to games. Afterward, the collected information is analyzed statistically, exploring the characteristics of teenagers addicted to digital games. Parents and teachers have the most contact with teenagers and know them the best, and game education professionals are authorities in digital games. Hence, a temporary team consisting of surveyed parents, teachers, and game education professionals is invited to put forward suggestions for improving the initially designed questionnaire. Then, researchers revise the questionnaire and determine the final draft.

The article "Electronic Sports Sustainable Development of Probing into Digital Games, Teenage Domestication, and Mutual Construction" was published in 2022. Journal: J Environ Public Health.

Answers available on the questionnaire include “excellent,” “acceptable,” “moderate,” “bad,” and “very bad,” scoring 5, 4, 3, 2, and 1 point, respectively. Using the SPSS 21 statistical analysis tool, the summed score of all questions represents the strength of the respondent's attitude. The Cronbach's *α* coefficient of this questionnaire survey is 0.805, exceeding 0.8, indicating its excellent reliability. Evaluated by a professional team, this questionnaire survey has a validity score lying between 0.79 and 0.98. The questionnaire survey is only for academic purposes and is performed with the consent of participants. No privacy information of the participants is disclosed, which confronts the standards and requirements of scientific research. The questionnaire is distributed via online (“Wenjuanxing”) and offline approaches. A total of 600 questionnaires were distributed, and 574 valid copies were returned, with a response rate of 95.7%. Therefore, the research objects were 574 students.

#### 2.5.2. Sampling of Questionnaire Survey

Second-order cluster sampling is adopted. First, schools are taken as the sampling units. One primary school, one junior high school, and one senior high school from Nanchang and Huaqiao are selected. Then, the sampling units are narrowed to classes. One class is selected, respectively, from the fourth and fifth grades of the primary school, the first and second grades of the junior high school, and the first and second grades of the senior high school. Finally, 574 teenagers from 5 schools in Nanchang and Huaqiao are included in the survey, including one primary school, one junior high school and one senior high school in Nanchang and one primary school and one senior high school in Huaqiao (including both junior and senior high schools).

Data and analysis results presented in any form during the interview and questionnaire survey are only the academic purposes, and no private information of the participants is disclosed, which confronts the standards and requirements of scientific research. The entire process of interview and questionnaire survey is the same for teenagers, parents, teachers, and game education professionals.

### 2.6. Result Analysis

The mutual domestication process and interactive relationship between teenagers and digital games are analyzed based on the interview and questionnaire survey results, including the contact with games, game guidance, game addiction, supervision, and game literacy and education.

The article "Electronic Sports Sustainable Development of Probing into Digital Games, Teenage Domestication, and Mutual Construction" was published in 2022. Journal: J Environ Public Health.

## 3. Results

### 3.1. Possession: Using and Distribution of Games

#### 3.1.1. Interview Results

Factors affecting teenagers' dominance of gaming equipment are age, academic results, and family atmosphere. Age is the most essential factor that affects the authority and quantity of teenagers' gaming equipment. “She is in the fourth grade, too young to own the electronic device” (Parent 1). “My son is in the sixth grade not separately, but the computer, tablet, and my mobile phone will be given to him to play” (Parent 4). Most parents do not allow teenagers to have their own electronic devices; nevertheless, teenagers are admitted with “temporary authority.”

The factor that ranks the second is academic results. Parents believe that games can affect teenagers' academic results, so electronic devices without gaming functions become the first choice. “When she was a child, her eyesight was damaged because of playing smartphones. Now, she is in high school and cannot play games” (Parent 6). “She was in junior high school with average grades. I equipped her with a phone watch, which can only be used to answer calls and cannot play games” (Parent 3). The third factor is the family atmosphere. If parents are game enthusiasts or their children have excellent academic results and strong self-control abilities, they will be more tolerant of electronic devices or games than other parents. “I do not have a desktop or a tablet. I go to the cybercafe to play games. My son and daughter use the old mobile phones of our families” (Parent 2). “My son is on the second day of junior high school, the top 10 in his class. He played games when he was a kid, and he does not play them now. Sometimes he checks WeChat to read the Ball Player with my phone” (Parent 5).

#### 3.1.2. Questionnaire Survey Results

Self-factors of teenagers' willingness to play games are considered. Demographics have affected the proportion of gamers among teenagers. There are 459 gamers out of 574 teenagers, accounting for about 80.0%. Gender and grade also influence the proportion of gamers. That of boys is 24.3% higher than that of girls. The proportions of gamers in primary school, junior high school, and senior high school students are 78.2, 86.9, and 74.5%, respectively, with the junior high school ranking the highest. Places of growth and academic results are critical influencing factors as well. The proportion of gamers among rural teenagers is 6.4% higher than that of urban teenagers. The proportion of gamers among students with good grades is 2.5% lower than that with moderate grades and 16.0% lower than that with poor grades.  Table 1 shows the details.

The article "Electronic Sports Sustainable Development of Probing into Digital Games, Teenage Domestication, and Mutual Construction" was published in 2022. Journal: J Environ Public Health.

To sum up, demographics greatly affect the proportion of gamers among teenagers, revealing the intrinsic motivation of gamers with different characteristics. Moreover, we have prepared a questionnaire to survey the 115 nongamers, in which the questions are multichoice, with four fixed options and one blank option that can be fulfilled by respondents themselves. The fixed options are “unable to purchase electronic devices due to economic reasons,” “strict parental supervision, with no access,” “playing games harms learning, which is emphasized at schools,” and “personal reasons, uninterested in playing games.”

Statistics suggest that, in terms of gender, reasons for not playing games are “strict parental supervision” and “personal reasons,” accounting for the same proportion among boys (40.0%). The uttermost reason for female nongamers is “personal reasons” (77.8%), followed by “strict parental supervision” (22.2%). Therefore, boys are more likely to own electronic devices and are regulated by parents.

Teenagers' grades are proportional to “personal reasons” (48.7% in the primary school, 53.8% in the junior high school, and 90.0% in the senior high school) and inversely proportional to “strict parental supervision” (41.0% in the primary school, 34.5% in the junior school for, and10.0% in the senior high school). With improved grades (increased age), parents admit more autonomy to teenagers with stronger self-control abilities.

The majority of urban and rural nongamers choose “personal reasons” (69.4% among the urban nongamers and 69.8% among the rural nongamers). The second-largest reason for nongamers is “strict parental supervision”; those who choose this reason in the urban area are 6.4% more than the rural area. Furthermore, there are 8.3% more nongamers in the urban area who choose “playing games harms learning, which is emphasized at schools” than those in the rural area, and the gap between nongamers caused by “economic reasons” in the urban and rural areas is 7.8%. In summary, rural teenagers are economically disadvantaged, preventing them from owning electronic devices; on the contrary, their parental supervision and school education are relatively relaxed. They have little or no contact with digital games, which can be a reason that they are not interested in games.

Among nongamers with poor grades, those who choose “personal reasons” are the least (65.2% among nongamers with excellent grades, 69.7% among those with good grades, 74.5% among those with moderate grades, and only 50.0% among those with poor grades). In contrast, 21.7% of nongamers with excellent grades choose “playing games harms learning, which is emphasized at schools,” ranking the largest (9.8% of nongamers with moderate grades 9.8%, and 12.5% of nongamers with poor grades). “Strict parental supervision” is chosen mostly by nongamers with extreme grades (excellent grades 30.4%, poor grades 37.5%); those with ordinary grades who choose this option account for less (good grades: 27.3%; moderate grades: 21.6%). Teenagers with lower grades are eager to own electronic devices, while those with extreme grades (excellent and poor) receive much supervision from their parents. The proportion of gamers among teenagers with excellent grades is the lowest, and that among teenagers with poor grades is the highest, indicating that the former is more subject to the supervision of parents and teachers.

The article "Electronic Sports Sustainable Development of Probing into Digital Games, Teenage Domestication, and Mutual Construction" was published in 2022. Journal: J Environ Public Health.

### 3.2. Materialization: Game Representation and Guidance

Materialization analysis is based on interviews. Parents have reported the following cases: “She is not allowed to play games around us, but she plays her grandma's mobile phone at grandparents' home” (Parent 3). “She uses her grandpa's mobile phone to play games while he is distracted” (Parent 1).

Mobile media eliminate family borders, making it difficult for parents to supervise their children. Left-behind children are less supervised by their parents and guardians. Teacher 1 mentioned that “Students get together to play after school. Children in the city are better supervised by their parents than those in the countryside, while the latter is more rampant in playing games.” The classroom, a space with the moral significance of “mission tuition,” is more repulsive to digital games and more restrictive in space. Most interviewed teachers oppose teenagers playing digital games. They believe that the fast-food Internet culture and sensory-stimulating games have prevented students from learning. Teachers ban smartphones in schools because of their professional habits of preventing extra factors such as ringtones from disrupting classroom order. “If students are found playing mobile phones in class, they will be criticized first, then the phones will be confiscated, and parents will be notified” (Teacher 3).

Digital games present different styles, and teenagers can choose how to participate. Games favored by teenagers can show their habits, tastes, and values. Interview results suggest that most parents neither play games nor allow their children to play games. Therefore, the types of games adored by teenagers can reflect their personalities and preferences. “He picks games himself, and I cannot control his preferences. His father occasionally plays games, but they are not interested in the same games.” (Parent 4). “She plays the small games brought by the computer, such as Drops and Doll Rehandling” (Parent 1). This record further proves that teenagers' choice of games also reflects their personality and preferences.

The article "Electronic Sports Sustainable Development of Probing into Digital Games, Teenage Domestication, and Mutual Construction" was published in 2022. Journal: J Environ Public Health.

The interviewed game planner believes that, on the one hand, the content, participation means, and themes of game live-streaming are the dominant representations of players themselves. On the other hand, grasping the preferences provides a new path for domesticating digital games, cultivating the games aesthetics of teenagers. “Mobile games focus on pleasure, and console games seek interaction, sharing, and education. I raise the threshold by guiding children to play good games, which cultivates game appreciation skills to avoid touching unhealthy games” (game planner).

### 3.3. Integration: Game Addiction and Supervision

#### 3.3.1. Interview Results

Regarding game addiction, education to teenagers by external factors, including parents and teachers, is as follows. First, parents control the frequency and duration of game-playing. “Monday to Friday are not allowed to play, and you can play at the time specified on the weekend” (Parent 1). “I control the length of the game, and he must give me the tablet or mobile phone immediately as required” (Parent 4).

Parents who play digital games have different supervision strategies from those who do not. The former uses the gaming skills correctly. They make full use of the “parent monitoring platforms” and “game antiaddiction systems” provided by developers to supervise the game-playing frequency and duration of their children. “My children and I team up to play the “Glory of the King.” If their academic performance improves, I buy the skins and props as rewards. However, they are strictly forbidden to play during their homework and school hours. I can notice whether they are secretly online” (Parent 2). In contrast, parents who do not play digital games may not understand the games well, making it easier for their children to “take advantage” in monitoring game frequency and duration. Besides, the lack of education in Internet security and the protection of gaming rights and interest cannot help teenagers cope with property theft and privacy leaks. “I do not play games, so I cannot deal with account theft or game fraud, but let him stop playing” (Parent 4).

Third, the imbalanced urban and rural educational resources affect the game guidance provided to teenagers. Public education places such as libraries, science and technology centers, and youth activity centers are abundant in cities. There are also more media and game literacy activities in schools and communities. Parents may seek help from professional game training institutions or psychological counseling centers to treat the game addiction of their children, which is disadvantageous for teenagers living in rural settings. “Game programming courses are provided in primary schools in first-line cities” (the teenager programming teacher). “Teenagers participate in various training, including dance, painting, aeromodelling, 3D printing, and badminton, which broadens their horizons and talents. Providing a place for teenagers in winter and summer vacations can prevent them from spending too much time on online games” (the teacher of an extracurricular activity center for teenagers).

The article "Electronic Sports Sustainable Development of Probing into Digital Games, Teenage Domestication, and Mutual Construction" was published in 2022. Journal: J Environ Public Health.

#### 3.3.2. Questionnaire Survey Results

Thirty-three of the 574 teenagers surveyed are addicted to games, accounting for 5.7%.  Table 2 proves that gender, grades, places of growth, academic results, and playing ages affect the percentage of game addiction. Specifically, 3.3% of the girls are addicted to games, while this rate among boys is 8.0%, 2.4 times that of the girls. The rates of game addiction in primary school, junior high school, and senior high school are 1.7%, 5.0%, and 10.2%, respectively, indicating that game addition is proportional to the grade. The rate of game addition among urban teenagers is 3.4%, and that among rural teenagers is 7.7%; the latter is 2.3 times the former. Moreover, the rates of game addition among teenagers with excellent, good, moderate, and poor grades are 1.3%, 4.3%, 6.7%, and 12.5%, respectively, showing that the worse the grade, the higher the addiction rate. The game addition rates among teenagers who have never played digital games, played for less than 2 years, played for 2–4 years, and played for more than 4 years are 0.0%, 3.8%, 8.8%, and 11.4%, respectively, revealing a proportional relationship.  Table 2 shows the details.

Data in Table 2 above reveal that the higher the frequency and the longer the playing periods, the more addicted the teenagers are. The places of growth, academic results, and whether they are left-behind children affect the proportion of game addiction. However, the main factors are the convenience of teenagers' access to games and the strictness of supervision by parents and teachers.

### 3.4. Transformation: Game Literacy and Education

#### 3.4.1. Interview Results

“The information technology courses in primary and secondary schools are limited to one course per week, which is difficult to add new content” (Teacher 4). “It is difficult to set up courses unrelated to the NCEE under the test-oriented education model. Students lack motivation” (Teacher 3). “I think that schools need to teach, but parent-assisted linkage cooperation has a good effect” (Teacher 5).

The article "Electronic Sports Sustainable Development of Probing into Digital Games, Teenage Domestication, and Mutual Construction" was published in 2022. Journal: J Environ Public Health.

Furthermore, parents equate “game literacy” with “game self-control consciousness” and expect schools to assume educational responsibilities for the lack of game literacy. “Never heard of “game literacy,” I think it is the self-control of games. The school teachers should teach it. We are nonplayers and do not know how to teach” (Parent 3). “We expect teachers to be strict and guide her to play healthy games” (Parent 1). In general, the educational abilities of families and schools for game literacy are far from each other's expectations. Therefore, not only teenagers but also parents, teachers, and the general public need to make up for game literacy lessons.

#### 3.4.2. Correlation Analysis

With control variables, a partial correlation analysis is made on the relationships among game technical ability, literary accomplishment, overall literacy, and game addiction.  Table 3 summarizes the analysis results. There is a positive correlation between game technical ability and game addiction, with a correlation coefficient of 0.246 (*P*=0.001 < 0.05). However, game literary accomplishment and overall literacy are negatively correlated to game addiction; the correlation coefficients are −0.522 (*P*=0.001 < 0.05) and −0.179 (*P*=0.001 < 0.05), respectively.

The above data concretely embody the mutual domestication of digital games and teenagers. On the one hand, the technical intention of digital games requires players to possess media knowledge and capabilities. The time of participation and the degree of involvement is positively correlated to the players' game technical ability. Also, the higher the technical ability of teenagers, the more likely they are addicted. Besides, players are familiar with the “routines” of media technology. They resist game addiction and restore control of the media by changing the strategies and reflecting on the media environment and information.

## 4. Discussion

The questionnaire survey suggests that digital games are often “controlled” and “uglified” in teenagers' lives. Parents and teachers participate in the domestication of games by teenagers and affect the results. Meanwhile, digital games have changed the way teenagers integrate into society. Electronic devices are the foundation for mutual domestication between digital games and teenagers, supported by the Research Report on the Behavior and Protection of Chinese Teenagers' Online Games. However, teenagers often use their parents' devices, while the dependence decreases with age [25]. Parents' intervention significantly influences the mutual domestication between teenagers and games. Demographics affect the proportion of gamers among teenagers. There are more gamers among boys than girls and more in rural area than in cities. As teenagers grow up, the proportion of gamers falls after rising. The proportion of gamers among teenagers with excellent grades is low, while that of teenagers with poor grades is high. Teenagers of different genders and ages enjoy different games, showing their unique styles, tastes, and values. Digital games are self-representations of teenagers. The sandbox game “Minecraft” [26], with 71.1% of the audiences aged 18 and below, ranks the first, followed by the casual mobile game “Battle of Balls” (53.0%). According to the 2018 iResearch, the primary audiences of multiplayer online games “League of Legends” and “Player unknown's Battlegrounds” aged 19–25, while the proportion of audiences aged 18 and below was 18.2 and 17.0%, respectively.

The article "Electronic Sports Sustainable Development of Probing into Digital Games, Teenage Domestication, and Mutual Construction" was published in 2022. Journal: J Environ Public Health.

Parents and teachers supervise teenagers playing digital games. Parents control the gaming equipment, time, and frequency of teenagers; teachers regulate the game behaviors by controlling the game location and time slot. Parents who play digital games or have good educational abilities take very different supervision strategies from those do not or have not. The unbalanced educational resources for game supervision in urban and rural areas result in the challenges of supervising the left-behind children. Teenagers with different characteristics have varying acceptance degrees of game supervision education from parents and teachers. For example, those with excellent grades have higher acceptance levels than those with poor grades.

Digital games affect the rhythm of teenagers' lives. In a positive perspective, teenagers can relax and form their social circles via games. Using the interaction and social features, teenagers can establish new social relations in the online community, correcting offline interpersonal relationships and peer friendship. Negatively, teenagers are prone to game addition. The portability and personalization of mobile media are not conducive to family supervision. Communication scholars who study the Internet or game addiction attach importance to the placement of home game devices. They suggest that parents keep computers in a place open to all members to monitor children's game behaviors [27]. If teenagers cannot control themselves or stop playing games on their own initiative, they will suffer from game addition. Integration analysis involves the time rhythm and usage habits of technology. Huazhen Zhou Research Group of the University of Chinese Academy of Social Sciences (UCASS) released the Survey Report on Adolescent Addiction Behavior, pointing out that Chinese teenage gamers who spend “1 day,” “2-3 days,” “4-5 days,” and “7 days” on digital games per week accounted for 17.5%, 21.5%, 5.9%, and 17.7% of the total. On a daily basis, the proportions of those who spend “1 hour,” “2-3 hours,” “4-5 hours,” “6-7 hours,” and “8 hours and above” on digital games are 51.1%, 30.9%, 9.3%, 3.2%, and 5.5%, respectively. The research group also claimed that teenagers who were addicted to games played digital games more than five days a week and five hours a day. Nearly one-fifth of teenagers in China are under the risk of game addiction [28].

The article "Electronic Sports Sustainable Development of Probing into Digital Games, Teenage Domestication, and Mutual Construction" was published in 2022. Journal: J Environ Public Health.

Game literacy education is an effective approach to prevent reverse domestication of technology [11, 29]. We have proved gaming literacy's resistance to game addiction through a questionnaire survey, revealing good gaming literacy of Chinese teenagers on the whole [30]. However, interviews reveal the insufficient game literacy of parents and teachers, whose educational abilities are far from each other's expectations. Families and schools face practical problems in teenagers' game literacy education.

## 5. Conclusions

We have analyzed the questionnaire and interview results comprehensively to investigate how digital games affect teenagers' physical and mental development and analyze the interactions and communications between teenagers and digital games [31]. Results demonstrate that gender, age, places of growth, and academic results can affect the proportion of gamers among teenagers. Games adored by teenagers can reveal their personalities and preferences. Parents and teachers supervise the time and frequency of teenagers playing games, and most of them hold an opposite attitude. Digital games greatly influence teenagers' lives; relaxation is a positive side, while addiction is a negative outcome [32]. Game literacy education can prevent reverse domestication effectively; however, its implementation still faces various challenges [33,34]. The research results provide a good idea for exploring the mutual domestication between teenagers and digital games, which are supported by specific qualitative and quantitative data.

This study has several limitations such as the questionnaire sampling is limited and it only comes from Jiangxi Province, which may not be enough to comprehensively represent the domestication relationship between teenagers and digital games. Some theoretical framework, game addiction, can be discussed with more details such as the causes and how to avoid addiction in adolescents. These two limitations will be improved in future works.

## Figures and Tables

**Table 1:** The proportion of gamers among teenagers of different genders, places of growth, grades, and academic results (the value represents the game-playing frequency).

Genders	Female (*N* = 299)	Male (*N* = 275)		

	67.3%	91.6%		
	*x* ^2^ = 53.086, df = 1, *P*=0.000			
Places of growth	Urban (*N* = 264)	Rural (*N* = 310)		
	76.5%	82.9%		
	*x* ^2^ = 3.632, df = 1, *P*=0.057			
Grades	Elementary school (*N* = 179)	Junior high school (*N* = 199)	High school (*N* = 196)	
	78.2%	86.9%	74.5%	
	*x* ^2^ = 10.045, df = 2, *P*=0.007			
Academic results	Excellent (*N* = 76)	Good (*N* = 188)	Moderate (*N* = 254)	Poor (*N* = 56)
	69.7%	82.4%	79.9%	85.7%
	*x* ^2^ = 6.841, df = 3, *P*=0.077			

The article "Electronic Sports Sustainable Development of Probing into Digital Games, Teenage Domestication, and Mutual Construction" was published in 2022. Journal: J Environ Public Health.

**Table 2:** Numbers and proportions of teenagers with different characteristics of game addiction.

Sample characteristics	Number of samples (*N* = 574)	
	Number of samples addicted	Addiction rate
Genders		
Male	24	8.0%
Female	9	3.3%
Grades		
Primary school	3	1.7%
Junior high school	10	5.0%
Senior high school	20	10.2%
Places of growth		
Urban	9	3.4%
Rural	24	7.7%
Results		
Excellent	1	1.3%
Good	8	4.3%
Moderate	17	6.7%
Poor	7	12.5%
Playing ages		
Never played	0	0.0%
Within 2 years	8	3.8%
2–4 years	11	8.8%
More than 4 years	14	11.4%

**Table 3:** Partial correlation coefficients between game technical ability, game literary accomplishment, game literacy, and game addiction.

Control variables	Analysis of item	
		Game addiction

Genders, grades, and playing periods	Game technical ability	*r* = 0.246, df = 569, *P*=0.001
Grades, results, places of growth, and playing periods	Game literary accomplishment	*r* = − 0.522, df = 568, *P*=0.001
Genders, grades, places of growth, and playing periods	Game literacy	*r* = − 0.179, df = 568, *P*=0.001

## Data Availability

The data used to support the findings of this study are available from the corresponding author upon request.

## References

[1] Bahremandpour A., Sheikholeslami S. M., Volkmann L. (2017). Roman game domination number of a graph. *Journal of Combinatorial Optimization*.

[2] Wong I. L. K., Lam M. P. S. (2016). Gaming behavior and addiction among Hong Kong adolescents. *Asian Journal of Gambling Issues & Public Health*.

[3] Sadat-Shirazi M. S., Vousooghi N., Alizadeh B. (2018). Expression of NMDA receptor subunits in human blood lymphocytes: a peripheral biomarker in online computer game addiction. *Journal of Behavioral Addictions*.

[4] Lin D., Bezemer C. P., Zou Y., Hassan A. E. (2019). An empirical study of game reviews on the Steam platform. *Empirical Software Engineering*.

[5] Kowert R. (2020). Dark participation in games. *Frontiers in Psychology*.

[6] Pallavicini F., Ferrari A., Mantovani F. (2018). Video games for well-being: a systematic review on the application of computer games for cognitive and emotional training in the adult population. *Frontiers in Psychology*.

The article "Electronic Sports Sustainable Development of Probing into Digital Games, Teenage Domestication, and Mutual Construction" was published in 2022. Journal: J Environ Public Health.

[7] Chen J., Ni P., Li X. (2018). Population size may shape the accumulation of functional mutations following domestication. *BMC Evolutionary Biology*.

[8] Siles L. (2019). The mutual domestication of users and algorithmic recommendations on netflix. Communication. *Cultural Critique*.

[9] Bonchev G., Dusinsky R., Hauptvogel P., Svec M. (2017). Patterns of evolutionary trajectories and domestication history within the genus hordeum assessed by REMAP markers. *Journal of Molecular Evolution*.

[10] Pan Z. D. (2014). Fun my iPhone, mess up my world Discuss the mediating and domesticating in the application of new media technology. *Journal of Suzhou University*.

[11] Liu Q. C., Zhang S. H. (2018). From tool to instinct repression: the phenomenon of reverse domestication in the era of intellectual media. *News Lovers*.

[12] Li B., Du X. H. (2016). Reverse domestication: a study on the influence mechanism of social media use and dependence on procrastination behavior taking University. *Students in Beijing as an example*.

[13] Liu T. Y. (2018). Analysis of the influence of social media on the academic performance of rural youths: taking the experience of X Village in Guanzhong Plain as an example. *Chinese Youth Research*.

[14] Goulden M. (2019). Delete the family: platform families and the colonization of the smart home. *Information, Communication &Society*.

[15] Fang L., Gong H., Hu Y. (2017). Genomic insights into divergence and dual domestication of cultivated allotetraploid cottons. *Genome Biology*.

[16] Ask K., Sørensen K. H. (2019). Domesticating technology for shared success: collective enactments of World of Warcraft. *Information, Communication & Society*.

[17] Han J., Du T., Zhang C., Qian X. (2018). Correlation analysis of CO2 emissions, material stocks and economic growth nexus: evidence from Chinese provinces. *Journal of Cleaner Production*.

[18] Wang Y. (2015). *Alternative Public Domain? Review of The Online Gaming Community*.

[19] Darvenkumar T., Anitha Devi V. (2022). A review on the impact of using E-games for social development and language acquisition in the English classroom. *ECS Transactions*.

[20] Big database of China Business Industry Research Institute (2019). *GDP Ranking of Provinces and Cities in the First Half of 2019*.

[21] Zhang W., Zhou H. (2019). *China Education Index*.

[22] Smith A., Pennington A., Carter B. (2018). Acceptability of the method of administration of a patient-reported outcome measure (PROM) with stroke survivors, a randomised controlled trial protocol. *Trials*.

The article "Electronic Sports Sustainable Development of Probing into Digital Games, Teenage Domestication, and Mutual Construction" was published in 2022. Journal: J Environ Public Health.

[23] Tencent (2019). *Ranking of China’s ‘Work Output’: Jiangxi Ranks Third, with the Champion’s Annual Outflow of 13 Million People*.

[24] Hameed U. A., Al-Jarrah M. D., Manzar M. D. (2020). Leeds sleep evaluation questionnaire in Jordanian university students. *Saudi Medical Journal*.

[25] Tencent Research Institute and DCCI Internet Data Center (2017). *Research Report on the Behavior and Protection of Chinese Youth Online Games*.

[26] Meng Q. (2017). Sandbox game <Minecraft> settled in China. *Computer Networks*.

[27] Chuang T. Y., Tsai C. M. (2015). Forecast the sarcity of game generation: digital game literacy. *New Media and Learning in the 21st Century*.

[28] Huazhen Z. (2018). *“Research Report on Teenagers’ Addictive Behavior: Based on the Data Analysis of 2017/2018 Youth Health Behavior Online Questionnaire,”*.

[29] Shen C. W., Min C., Wang C. C. (2019). Analyzing the trend of O2O commerce by bilingual text mining on social media. *Computers in Human Behavior*.

[30] Chen M. (2018). The research of human individual’s conformity behavior in emergency situations. *Library Hi Tech*.

[31] Chen M. (2019). The impact of expatriates’ cross-cultural adjustment on work stress and job involvement in the high-tech industry. *Frontiers in Psychology*.

[32] Liu Y., Chen M. (2018). From the aspect of STEM to discuss the effect of ecological art education on knowledge integration and problem-solving capability. *EKOLOJI*.

[33] Feng B., Chen M. (2020). The impact of entrepreneurial passion on psychology and behavior of entrepreneurs. *Frontiers in Psychology*.

[34] Zheng Y., Zhou Y., Lai Q. (2015). Effects of twenty-four move shadow boxing combined with psychosomatic relaxation on depression and anxiety in patients with type-2 diabetes. *Psychiatria Danubina*.

